RETRACTED

# Psychosocial Factors and Psychological Characteristics of Personality of Patients with Chronic Diseases Using Artificial Intelligence Data Mining Technology and Wireless Network Cloud Service Platform

**DOI:** 10.1155/2022/8418589

**Published:** 2022-04-13

**Authors:** Kangqi An

**Affiliations:** School of Psychological and Cognitive Sciences, Peking University, Beijing 100871, China

## Abstract

It was to explore the application value of health cloud service platform based on data mining algorithm and wireless network in the analysis of psychosocial factors and psychological characteristics of personality of patients with chronic diseases. Based on the demand analysis of cloud service platform for chronic diseases, a health cloud service platform including three modules was established: support layer, application layer, and interaction layer; and K-means algorithm and Apriori algorithm were used to mine and process data. The changes of pulse wave and EEG signal of epileptic seizures before and after processing by wireless network health cloud service platform were analyzed. 42 patients with idiopathic generalized epilepsy were selected as the research subjects, and 40 volunteers with normal physical examination during the same period were selected as the control group. The differences in the basic clinical characteristics data, Hamilton Anxiety Scale (HAMA), Hamilton Depression Scale (HAMD), Symptom Checklist 90 (SCL-90), and Eysenck Personality Questionnaire-Revision Short Scale for Chinese (EPQ-RSC) were compared between the two groups. It was found that the initial EEG signals of epileptic patients had noise pollution before and after the seizure, and the noise in the EEG signals was filtered out after digital technology processing in the cloud service platform. The maximum number of epileptic patients aged 18∼30 years was 17 (40.48%), and the mean scores of HAMD and HAMA scales in the epileptic group were significantly higher than those in the control group (*P* < 0.001). The total score of SCL-90, somatization, obsessive-compulsive symptoms, interpersonal sensitivity, depression, anxiety, hostility, phobic anxiety, paranoid ideation, and psychosis in the epilepsy group were obviously higher than those in the control group (*P* < 0.01). The mean value of EPQ-RSC and neuroticism (*N*) was clearly higher (*P* < 0.05), the mean value of extroversion (*E*) was significantly lower (*P* < 0.01), and the mean value of Lie Scale was significantly higher (*P* < 0.05) in the epileptic group in contrast with those in the control group. It indicates that the cloud service platform for chronic diseases based on artificial intelligence data mining technology and wireless network has potential application value. Epilepsy patients with chronic diseases should be paid more attention to their psychosocial factors and psychological characteristics of personality in the treatment process.

RETRACTED

## 1. Introduction

Dynamic environment is the difference in form, connotation, and state of the consistency of macroeconomic environment, industrial environment, internal environment, external environment, and social environment with the change of time. Among them, various environments are in a complex and variable state of change and instability. The main feature of dynamic environment is change [1]. With the rapid development of social economy and the change of people's lifestyle, the diseases threatening human health are gradually changed from infectious diseases to noncommunicable diseases (NCDs). A survey report by the World Health Organization (WHO) pointed out that NCDs have become the primary factor of human death [2]. The main harm of NCDs is to cause damage to important organs such as heart, brain, and kidney, and lifelong diseases [3]. According to statistics, the incidence of NCDs such as diabetes, cardiovascular disease, chronic respiratory disease, and cancer has been increasing year by year in recent years. The results of some studies and statistics indicated that the total number of chronic diseases has exceeded 260 million worldwide, and the total cost of NCDs accounts for about 70% of the total health cost, which is even as high as 73% in 2020 [4]. Therefore, NCDs have a serious impact on human quality of life and economic burden and have become an important public health problem. With the development of “biopsychosocial medical model,” more and more people pay attention to psychosocial factors, psychological characteristics of personality, and the occurrence of diseases. Biological factors and nonbiological factors are the main factors affecting human health, with nonbiological factors being also known as psychosocial factors, including psychological factors and social factors [5]. Psychological factors refer to personality traits and emotional states that affect human health. Social factors refer to the living and working environment. With the improvement of people's living standards and the progress of medical technology, in the process of diagnosis and treatment of diseases, not only the impact of biological factors on people, but also the impact of psychological and social factors on health is considered [6]. Personality is an individual's internal tendency in behavior, which is manifested as the integration of ability, emotion, need, motivation, interest, attitude, values, temperament, personality, and physique when an individual adapts to the environment. It is self-dynamic consistency and continuity, which makes the individual form a characteristic psychosomatic organization in the process of socialization [7]. Social psychological factors and psychological characteristics of personality in different age, occupation, and social class can get different stress [8]. Some studies have pointed out that patients with chronic diseases are prone to produce more psychological symptoms and more psychological problems and have a certain degree of influence on the development and prognosis of the disease. Different psychological and social factors and psychological characteristics of personality of patients with different chronic diseases lead to different stress on the immune system [9]. At present, studies have presented that patients with chronic diseases such as cancer, chronic cheilitis, burning mouth syndrome, metabolic syndrome, hypertension, and diabetes have different degrees of psychological problems [10].

RETRACTED

Information, as a valuable resource of modern enterprises, occupies an increasingly important position. It has become the basis of scientific management of modern enterprises, the premise of correct decision-making, and the means of effective regulation. The Internet, wireless, and communication networks are the two core products of the new era. Mobile phones and computers have become “necessities” in people's lives. With the emergence of cloud computing and the maturity of 3G wireless communication networks, the handover of cloud computing and wireless network technology has become a new research hotspot [11]. Under the background of “Internet +”, big data plays an important role in disease monitoring, auxiliary decision-making, health management, and other fields and is the key trend of the development of smart medicine in the future [12]. The application of digital technology (DT) in clinical medicine mainly involves the processing of medical image, electrophysiological signal, and other information generated by digital medical equipment and rehabilitation treatment equipment [13]. On the other hand, the application of DT in the medical field also involves processes such as the collection, intelligent processing, and management of medical big data [14]. As the basic medical data of DT, medical informatization is derived from the clinical and monitoring data of hospitals, research data of medical scientific research institutions, and self-health data directly collected by individuals [15]. Using cloud computing as the basis of medical data mining platform can not only effectively solve the problem of recording and storing medical data, but also provide the basis for the analysis and calculation of medical data [16]. The health cloud service platform is to transmit the health data collected by digital general practice diagnostic equipment to the cloud data center, integrate personal basic medical information, and provide personal-centered health management, diagnosis, and early warning services for community residents and their families, so as to realize the combination of Internet technology and general practice diagnostic equipment [17]. The health cloud platform realizes remote real-time monitoring of user health status through the collection, processing, and analysis of user health data, providing a guarantee for medical big data storage and analysis [18]. Data mining is developed through various technical theories and user needs. Machine learning, database, and statistics are the key technologies of data mining [19]. However, the current DT-based health cloud platform focuses more on data acquisition and data visualization display, and there is a lack of further analysis and mining of user health data [20].

RETRACTED

In summary, there are few studies on the analysis of psychosocial factors and psychological characteristics of personality of patients with chronic diseases, and the current DT-based health cloud platform lacks the analysis and mining of user health data. Therefore, this study analyzes and mines the relevant data of psychosocial factors and psychological characteristics of personality of patients with chronic diseases based on DT health cloud platform, summarizes those, fully grasps the psychological conditions of patients while performing symptomatic treatment, and provides a reference direction and certain guiding significance for correct counselling and guiding the psychology of patients.

## 2. Materials and Methods

### 2.1. Structure of Health Cloud Service Platform for Chronic Diseases

Requirement analysis is the primary solution to project development and design [21]. The requirements of health cloud service platform generally include four aspects: business needs, user needs, functional needs, and nonfunctional needs. Among them, the business needs are the basis of the cloud service platform. Combined with the current development status of medical cause in China, the business needs of the health cloud service platform mainly involve three aspects: patients, medical staff, and management. Community resident business includes health records, self-health management, health monitoring, and health early warning. User needs mainly include the types of medical service providers and the specific needs of patients. The functional requirements determine various services that the platform can provide, including user login, registration, personal information storage, health data monitoring results, diagnosis and treatment information inquiry, and health consultation information push. Nonfunctional needs are the judgment of platform adaptability, reliability, and maintainability. The demand analysis structure of health cloud service platform based on chronic diseases is illustrated in Figure 1.

RETRACTED

Based on demand analysis, the chronic disease health cloud service platform is mainly composed of support layer, application layer, and interaction layer modules. The support layer is mainly the storage of various types of data, the deployment of cloud service platform, and user operation environment. In terms of data storage, the relational database MySQL is used for data structuring, and for unstructured types of data, the HBase database [22] is adopted for storage. The deployment environment is supported by the Web application server Tomcat [23], and the operation environment selects a commonly used web browser to provide the user with a use interface. The application layer realizes the health service needs of upper users through engineering design, which is mainly composed of three parts: data layer, key technology layer, and functional module layer; the interaction layer mainly communicates data with the application layer and presents the information management system of various services to the users, and its main task is to provide the users with the health-related medical application services they need. The application layer responds to the requests made by the interaction layer through database query and analysis and returns them to the interaction layer for users to view and use. The basic framework of the chronic disease health cloud service platform is given in Figure 2.

Digital diagnostic equipment mainly includes commonly used blood pressure detection, blood glucose detection, blood oxygen saturation detection, pulse rate detection, body temperature detection, and electrocardiogram (ECG). The measurement results of height and weight can be obtained by wired or wireless connection. The measurement data are automatically digitally integrated with other data of patients, which can effectively reduce the working intensity of medical personnel and become an effective auxiliary tool for diagnosis and treatment of general practitioners. In terms of information collection, the detection parameters include general data such as height, weight, and body temperature, and special data such as blood pressure, blood oxygen, and ECG. In the process of parameter detection and acquisition, the nonlinear geometric feature filtering method is applied to filter out the noise and interference mixed with the detection signal on the waveform and spectrum. Database pattern matching algorithm is used to realize automatic matching between adaptive ECG template and patient ECG data. In the aspect of image processing, the integrated application of image segmentation, texture analysis, image registration, and image fusion technology, combined with digital signal processing and access optimization algorithm and ECG, blood oxygen waveform, and other real-time rendering algorithms, the medical imaging of the detection data is realized. The collected signal is processed by digital filtering. The physiological parameters are calculated based on the waveform signal, and according to the physiological parameters, preliminary pathological judgment is obtained. In order to further filter out the noise, the simulated sampling data is digitally filtered, and the physiological parameters such as heart rate and blood pressure can be calculated by combining various waveform signals, so as to carry out certain pathological judgment.

RETRACTED

The cloud computing framework is mainly composed of Hadoop distributed file system (HDFS), parallel programming model MapReduce, and distributed database HBase components. HDFS distributed file system is a master-slave structure system, with NameNode as the main node to manage the metadata of file system and DateNode as the slave node to store the actual data. MapReduce is a programming model for parallel computing of large-scale data sets. By distributing operations on large-scale data sets to each node under the management of a master node, the final result is obtained by integrating the intermediate results of each node. HBase is a distributed and extensible NoSQL database running on Hadoop. Its underlying storage support is HDFS file system, and MapReduce model is used to process the data stored in it. In addition, Zookeeper provides distributed coordination services such as centralized configuration management, grouping, and command for HBase.

### 2.2. Database Design of Chronic Disease Cloud Service Platform Based on DT

Health care data includes many types of data such as user information, index data, clinical test data, image pictures, pathological analysis, and video audio. The data layer contains various types of data and files. In this study, a database of chronic disease cloud service platform is established by combining vertical segmentation method, mainly including patient basic information, medical history, disease diagnosis, and evaluation index tables. The specific information in the database is shown in Tables 1–4.

### 2.3. Chronic Disease Data Mining of Cloud Service Platform Based on DT

Medical data are often diverse, incomplete, and random [24], so they need to be preprocessed before the process analysis of medical data. Data preprocessing mainly includes data selection and data transformation. The preprocessed data is further analyzed by data mining technology, and the data mining process mainly includes selective preparation of data, its analysis by appropriate mining algorithms, and finally interpretation and analysis of the mined results. The specific process of chronic disease data mining in cloud service platform based on DT is given in Figure 3.

RETRACTED

Data mining results mainly include two categories: descriptive analysis and predictive analysis [25]. Descriptive analysis groups the mined data according to the similarity between the data and obtains the potential laws implied in the data, mainly including cluster analysis and association analysis. Clustering is to classify the data records with similar attribute characteristics in the dataset and, at the same time, divide the data with large difference in attribute characteristics into different categories. K-means algorithm is a commonly used cluster analysis tool in data mining [26]. It is supposed that there are *n* records for medical data mining results, and each record selects *l* variables, then the measurement value of the *k*th variable of the *i*th record is *a*_*ik*_, and the data matrix of this sample can be expressed as follows.

(1) $$\begin{array}{c} A=\left[\begin{array}{c} a_{11\;}a_{12}\cdots a_{13}\\ a_{21\;}a_{22}\cdots a_{23}\\ \vdots \vdots \cdots \vdots \\ a_{n1\;}a_{n2}\cdots a_{n3} \end{array}\right]. \end{array}$$

The mean of the *k*th variable can be expressed as follows:

(2) $$\begin{array}{c} a_{ik}=\frac{1}{n\;}\overset{n}{\underset{i=1}{\sum }}a_{ik}. \end{array}$$

After centralization and standardization of mining data, *n* records of the *k*th variable can be expressed as equation (3) after centralization, and *n* records of the *k*th variable can be expressed as equation (4) after standardization, where *S*_*k*_ is the standard deviation of the *k*th variable.

(3) $$\begin{array}{c} {\tilde{a}}_{ik}=a_{ik}-{\bar{a}}_{ik}, \end{array}$$

(4) $$\begin{array}{c} a_{ik}^{\prime }=\frac{a_{ik}-{\bar{a}}_{ik}}{S_{k}}. \end{array}$$

The similarity between each record is measured by distance. For *l* variable records, *n* records can be regarded as *n* points in the *l* dimension space, and the distance between the *i*th record and *j*th record in the dataset can be expressed as follows:

(5) $$\begin{array}{c} d_{ij}\left(l\right)={\left[\overset{l}{\underset{k=1}{\sum }}{\left|a_{ik}-{\bar{a}}_{ik}\right|}^{l}\right]}^{1/l},l>0. \end{array}$$

The clustering analysis method based on K-means algorithm inputs the data set and the number of categories. After the initialization of the class center, the center distance is calculated, and the above steps are repeated according to the threshold classification until the criterion function converges, as well as the output category combination. The specific process of clustering analysis based on K-means algorithm is illustrated in Figure 4.

RETRACTED

Association rules reflect the interdependence and relevance between one thing and other things. The probability of simultaneous occurrence of item sets *M* and *N* is called the support of association rules, which is shown in the following equation:

(6) $$\begin{array}{c} S\left(\text{M}⟹\text{N}\right)=P\left(M\cap N\right). \end{array}$$

The confidence of association rules refers to the probability that item set *N* also appears when item set *M* appears, and its calculation method is as follows:

(7) $$\begin{array}{c} C\left(\text{M}⟹\text{N}\right)=P\left(\text{M}|\text{N}\right). \end{array}$$

Association rules related algorithms mainly include Apriori algorithm, FP-tree algorithm, and Eclat algorithm. Among them, Apriori algorithm is a classical algorithm for mining frequent item sets in association rules, which has obvious advantages in association rules [27]. For a given database *B*, its items set *E* and things set *T* are presented as follows:

(8) $$\begin{array}{c} \text{E}=\left\{E_{1,}E_{2\;},\;\cdots E_{m\;}\right\},\\ \text{T}=\left\{T_{1,}T_{2},\cdots T_{n}\right\}. \end{array}$$

The transaction Boolean matrix *F* of database *B* mapping is expressed as follows:

(9) $$\begin{array}{c} \text{F}=\left(f_{ij}\right)=\left\{\begin{array}{c} 1,E_{j}\in T_{i}\\ 0,E_{j}∄T_{i} \end{array}\right\},\text{i}=1,2,\cdots ,\text{n};\text{j}=1,2,\cdots ,\text{m.} \end{array}$$

*m* represents the number of items, and *n* is the number of transactions.

The vector of each item *E* in database *B* is presented in the following equations:

(10) $$\begin{array}{c} {\text{G}}_{i}=x_{i1,}x_{i2},\cdots x_{im},\\ x_{ij}=\left\{\begin{array}{c} 1,E_{j}\in T_{i}\\ 0,\;E_{j}∄T_{i} \end{array}\right\}. \end{array}$$

Each support technology is expressed as follows:

(11) $$\begin{array}{c} S\left(E_{i}\right)=\overset{n}{\underset{i=1}{\sum }}x_{ij}. \end{array}$$

### 2.4. Data of Chronic Disease Patients Based on Cloud Service Platform

A total of 42 patients (26 males and 16 females) with idiopathic generalized epilepsy who visited the epilepsy clinic of the Department of Neurology, Sanbo Brain Hospital Capital Medical University, from June 2019 to June 2021 were selected as the study subjects. The age of the patients ranged from 19 to 80 years; the mean age was 50.35 ± 4.85 years. The inclusion criteria of this study were as follows: patients with epilepsy diagnosed by 24-hour ambulatory electroencephalography and cranial imaging examination; patients older than 18 years; patients' duration of disease ≥1 year; patients having normal language expression and dictation ability and being able to independently complete the rating scale; patients not taking psychiatric related drugs within two weeks. Exclusion criteria: patients with severe cognitive and mental retardation; patients with intracranial lesions suggested by head CT or MRI; patients with other tumors; patients with severe dysfunction of important organs; patients with family history of mental illness; long-term use of other drugs and substance abusers other than antiepileptic drugs. Forty volunteers with normal physical examination during the same period were included as the control group, aged 19∼80 years. The inclusion criteria for the control group were as follows: patients with normal physical examination; patients without history of chronic diseases and mental illness; patients without family history of epilepsy. Exclusion criteria: patients taking psychiatric related medications are excluded. The trial procedures of this study were approved by the Ethics Committee of Sanbo Brain Hospital Capital Medical University, and the subjects included in the study signed an informed consent form.

RETRACTED

### 2.5. Analysis of Psychosocial Factors and Psychological Characteristics of Personality in Patients with Chronic Diseases

The psychological status of the patients was analyzed based on the Symptom Check List-90 (SCL-90) in the cloud service platform, which is mainly used to assess emotion, consciousness, thinking, behavior, and psychological status [28] and contains a total of 90 items and 9 factors. Each item adopts a 5-level scoring system. There are no symptoms, 1 point; subjective symptoms are very light, 2 points; subjective symptoms are general or moderate, 3 points; subjective symptoms are heavy, 4 points; subjective symptoms are severe, 5 points.

Hamilton anxiety scale (HAMA) [29] was used to assess the anxiety level of subjects. The HAMA scale includes two aspects: somatic anxiety and mental anxiety, with 14 items. All items were scored on a 5-level scale from 0 to 4. Total score >29 points, it may be severe anxiety; >21 points, it must have significant anxiety; >14 points, it must have anxiety; between 7 and 14 points, it may have anxiety; <7 points, no anxiety.

Hamilton depression scale (HAMD) [30] was used to assess the depression level of subjects. There was a total of 5 aspects and 17 items. Among them, 8 items of difficulty falling asleep, not deep sleep, early awakening, gastrointestinal symptoms, systemic symptoms, sexual symptoms, weight loss, and insight were scored on a 3-level scale of 0–2, and the remaining items were scored on a 5-level scale of 0–4. Total score >24 points, it is considered severe depression, >17 points, it is mild-moderate depression, between 7 and 17 points, it is probable depression, and <7 points, no depressive symptoms. The higher score, the more serious depressive symptoms.

RETRACTED

The personality characteristics of the patients were analyzed based on the Eysenck personality questionnaire-revised short scale for Chinese (EPQ-RSC) in the cloud service platform [31], and the EPQ-RSC had a total of 48 items, including four aspects: psychoticism scale (*P*), extroversion (*E*), neuroticism (*N*), and lie scale (*L*). For each item of EPQ-RSC (forward scoring), selecting “Yes”, 1 point, selecting “No” 0 point. Reverse score is opposite.

### 2.6. Statistical Methods

The test data were processed by SPSS 19.0 statistical software. The measurement data were expressed as mean ± standard deviation ($\bar{\text{x}}$ ± *s*). The enumeration data were expressed as percentage (%). The *χ*^2^ test was used. *P* < 0.05 indicated that the difference was statistically significant.

## 3. Results

### 3.1. Data Processing Results Analysis Based on DT Cloud Service Platform

ECG signal data is processed based on DT cloud service platform. The results suggest that the original collected pulse wave has a small amplitude oscillation at the trough, and there is obvious noise at the same time. The amplitude of pulse wave oscillation is apparently reduced after digital processing of cloud service platform, and the waveform noise has been filtered out (Figures 5 and 6).

The acquired EEG signal data of epileptic patients were processed based on the DT cloud service platform. The results showed that the initial EEG signal of epileptic patients had noise pollution before and after seizure. The noise in EEG signal was filtered out after digital processing of cloud service platform, which could better present the EEG signal of epileptic patients during seizure (Figures 7 and 8).

### 3.2. Basic Information of Included Subjects

The age of the subjects included in the study was statistically analyzed (Figure 9). The largest number of epilepsy patients aged 18–30 years was 17, accounting for 40.48%, followed by 31–40 years, a total of 10 (23.81%). The number of patients aged 61–70 years old was 7, accounting for 16.67%, and the number of patients aged 71–80 years old was at least 1 (2.38%).

Average age, gender, nationality, regional distribution, education level, occupation, and marital status of patients with epilepsy and the control group were further compared and analyzed (Table 5). There was no obvious distinction in the average age, gender, nationality, regional distribution, education level, occupation, and marital status between the observation group and the control group (*P* > 0.05).

RETRACTED

## 4. Comparison of HAMA and HAMD Scores of Included Subjects

The results of HAMA and HAMD scale scores in epileptic patients and control group were compared and analyzed (Figure 10). The mean value of HAMA score in epileptic patients was (7.51 ± 1.35), and the mean value of HAMA score in control group was (3.39 ± 0.98). The mean value of HAMA score in epileptic patients was significantly higher than that in control group, with very significant difference between the two groups (*P* < 0.001). The mean scores of HAMD scale in epilepsy group and control group were (5.68 ± 0.75) and (2.06 ± 0.28), respectively. The mean scores of HAMD scale in epilepsy group were significantly higher than those in the control group (*P* < 0.001).

### 4.1. Comparison of SCL-90 Scores

The results of SCL-90 scores between epilepsy patients and controls were contrasted and analyzed (Figure 11), and the mean total SCL-90 score was (2.58 ± 0.21) in epilepsy patients and (1.29 ± 0.10) in controls, and the mean total SCL-90 score in epilepsy patients was distinctly higher than that in controls (*P* < 0.01). The somatization score of epilepsy patients was (2.71 ± 0.22) and that of controls was (1.23 ± 0.09). The somatization score of epilepsy patients was distinctly superior than that of controls (*P* < 0.01). The obsessive-compulsive symptom score of epilepsy patients was (2.92 ± 0.23), while that of controls was (1.45 ± 0.11). The obsessive-compulsive symptom score of epilepsy patients was clearly higher in contrast with that of controls (*P* < 0.01). The result of interpersonal sensitivity was (2.37 ± 0.19) in patients with epilepsy and (1.28 ± 0.10) in controls. The interpersonal sensitivity score of patients with epilepsy was clearly superior versus that of controls (*P* < 0.01). The scores of depression, anxiety, hostility, phobic anxiety, paranoid ideation, and psychosis in patients with epilepsy were (3.05 ± 0.24), (2.64 ± 0.21), (2.26 ± 0.18), (2.19 ± 0.18), (2.08 ± 0.17), and (2.45 ± 0.20), respectively. The scores of those in controls were (1.87 ± 0.14), (1.24 ± 0.09), (0.77 ± 0.06), (0.71 ± 0.05), (0.63 ± 0.05), and (1.08 ± 0.08), respectively. The scores of depression, anxiety, hostility, phobic anxiety, paranoid ideation, and psychosis in patients with epilepsy were significantly higher than those in controls (*P* < 0.01).

RETRACTED

### 4.2. Comparison of EPQ-RSC Scale Scores

The results of EPQ-RSC scale scores between epilepsy patients and controls were compared and analyzed (Figure 12), and the mean value of psychoticism (*P*) scale was (3.59 ± 0.24) in epilepsy patients and (2.51 ± 0.17) in controls, and the mean value of EPQ-RSC psychoticism scale was apparently higher in epilepsy patients than that in controls (*P* < 0.05). The mean value of extroversion (*E*) was (5.33 ± 0.35) in patients with epilepsy and (8.89 ± 0.59) in controls. The mean value of extroversion of EPQ-RSC psychoticism scale in patients with epilepsy was apparently lower than that in controls (*P* < 0.01). The mean value of neuroticism (N) was (7.02 ± 0.46) in epilepsy patients and (3.74 ± 0.25) in controls. The mean value of neuroticism in EPQ-RSC psychoticism scale in epilepsy patients was obviously superior than that in controls (*P* < 0.01). The mean value of lie scale (*L*) was (5.74 ± 0.38) in epilepsy patients and (4.36 ± 0.29) in controls, and the mean value of lie scale in EPQ-RSC psychoticism scale was obviously superior in epilepsy patients versus that in controls (*P* < 0.05).

## 5. Discussion

In the diagnosis of human diseases, the diagnosis of human pulse wave plays an important role, and human pulse wave is important in the transmission of physiological and pathological information of a variety of diseases [32]. In order to verify the processing effect of cloud service platform based on DT on medical data, the collected pulse waves are processed in this study, and the results show that the pulse wave oscillation amplitude after DT processing of cloud service platform is reduced, and the waveform noise has been filtered out. The results reveal that the quality of pulse image is increased after digital processing of cloud service platform. Epilepsy is a chronic disease that affects the physical, emotional, and social life of patients [33]. Epileptic patients not only suffer from physical damage caused by seizures, but also face the adverse reactions caused by antiepileptic drugs, the pubic sensation caused by the disease, and the ensuing anxiety and depression, which seriously affect the quality of life of patients [34]. The EEG contains a large amount of physiological and pathological information, such as characteristic waves such as echoes and slow waves during seizures, so it plays a crucial role in epilepsy diagnosis [35]. Usually, about 80% of epileptic patients have abnormal information on the EEG, and if the EEG is appropriately induced, then 90% or more of epileptic patients will present with abnormal EEG [36]. The results of this study found that the initial EEG signal had noise pollution before and after the seizure, and the noise in the EEG signal was filtered out after the digital technology processing of cloud service platform, which could better present the EEG signal during the patient's seizure. This lays a foundation for subsequent data mining and data analysis.

RETRACTED

According to statistics, the incidence of depression in patients with recurrent epilepsy is 20%∼55% [37]. The age of the subjects included in this study was analyzed, and the results suggested that the maximum number of epileptic patients aged 18∼30 years in the included study was 17, accounting for 40.48%, followed by 31∼40 years, a total of 10 (23.81%). The incidence between 61 and 70 years was 7 cases, which accounted for 16.67%, and the minimum number of epileptic patients between 71 and 80 years was 1 case (2.38%). This is mainly due to idiopathic epilepsy, traumatic brain injury, infection, and epilepsy caused by congenital developmental malformations in young patients, symptomatic epilepsy caused by brain tumors and traumatic brain injury in middle-aged patients, and symptomatic epilepsy caused by cerebrovascular disease, brain tumors, and traumatic brain injury in elderly patients [38]. The results of current studies indicated that psychological factors play a role in the occurrence and development of chronic diseases and cancer [39], and some studies pointed out that adverse psychological factors can lead to changes in human endocrine and cranial neuromediators, which in turn decrease the body's immunity and ultimately lead to disease progression or cancer occurrence [40]. In addition, some researchers pointed out that, under psychological stress, the body's neuroendocrine-immune system changes, which has a certain impact on the process of tumor adhesion, proliferation, migration, and invasion, and then affects the occurrence and development of tumors [41]. Therefore, psychological factors play an important role in the development of chronic diseases and tumors.

With the proposal of biopsychosocial medical model, the treatment of epilepsy no longer only focuses on seizures and cognitive impairment, but also lies in improving the quality of life of patients and the analysis of psychosocial factors and personality and psychological characteristics. Comorbid depression in epilepsy is associated with genetic and psychosocial factors [42]. Comorbid anxiety in epilepsy may be related to psychosocial mechanisms and neuropathological mechanisms [43]. Studies have shown that depressive symptoms are a routine psychological response in patients with epilepsy and need not be given too much attention [44]. The results showed that the mean scores of HAMD and HAMA in the epilepsy group were obviously superior than those in the control group (*P* < 0.001). These results suggest that patients with epilepsy all have significant depression and anxiety. If it is not intervened, it will further affect the quality of life of patients. Therefore, in clinical work, while paying attention to the therapeutic effect of epilepsy patients, it must enhance the awareness of comorbidity of epilepsy and depression and anxiety, conduct routine screening of depression and anxiety for epilepsy patients [45], and carry out targeted psychological intervention to reduce the more profound impact of anxiety and depression on the life of epilepsy patients. Butler et al. [37] presented that patients with epilepsy are more susceptible to anxiety and depression than the normal population, and this emotion predisposes patients to distortion of their understanding of the disease, loss of confidence in treatment, more passive in interpersonal communication, reducing social activities, and alienation of family relationships, resulting in reduced social support, reduced subjective well-being, invisibly aggravating patients' anxiety and depression symptoms, and further reducing the quality of life.

RETRACTED

The SCL-90 scale has some scientificity and practicability in assessing the psychiatric symptoms or psychological status of the subjects from emotional, conscious, thinking, and behavioral aspects [46]. The results of SCL-90 scores in patients and controls were analyzed. The results indicated that the mean SCL-90 total score, somatization score, obsessive-compulsive symptom score, interpersonal sensitivity score, depression, anxiety, hostility, phobic anxiety, paranoid ideation, and psychosis scores in patients were visibly superior than those in controls (*P* < 0.01). Somatization is mainly used to assess patients' subjective physical discomfort symptoms, such as anxiety and headache. Obsessive-compulsive symptoms refer to the patient's behavior of knowing nothing but repeatedly doing something [47]. Interpersonal sensitivity refers to the fact that patients are often accompanied by low self-esteem, suspiciousness, and tension during communication with people [48]. Hostility is mainly evaluated from three aspects: thought, emotion, and behavior [49]. Paranoia is mainly the bad mood that patients show when they face others [50]. Current findings suggest that long-term adverse psychological emotions can have some impact on the body's immunity and ultimately affect the progression of cancer [51]. The results of this study are similar to those of the current study. The EPQ-RSC scale is mainly adopted to assess adult psychoticism, extroversion, neuroticism, and lie scales [52]. The results of this study revealed that the mean value of EPQ-RSC psychoticism scale in epilepsy group patients was obviously higher than that in controls (*P* < 0.05). The mean extroversion value of epilepsy group patients was obviously inferior than that of controls (*P* < 0.01), and the neuroticism and lie scales were higher than those of controls (*P* < 0.011). These results suggest that patients show high psychoticism and neuroticism, and they are more likely to be introverted. Some studies presented those patients show control of self-emotions, are not good at expression, and are introverted [53], and the results are similar to the studies.

RETRACTED

## 6. Conclusion

The psychosocial factors and psychological characteristics of personality of patients with chronic diseases (epilepsy group) were evaluated based on the digital technologized cloud service platform. The results showed that patients with epilepsy group had obvious psychological problems and introverted instability in personality and showed concealed personality to a certain extent. However, there are still some shortcomings in this study. This study only analyzes the psychosocial factors and psychological characteristics of personality of patients with epilepsy group but does not analyze other types of chronic diseases. In the future work, the psychosocial factors and psychological characteristics of personality of other chronic diseases will be analyzed based on the digital technologized cloud service platform established in this study, providing a more comprehensive reference for the diagnosis and treatment of chronic diseases. In conclusion, the chronic disease cloud service platform based on DT has potential application value, and more attention should be paid to psychosocial factors and psychological characteristics of personality during the treatment of patients with chronic diseases (epilepsy group).

## Figures and Tables

**Figure 1:** Structure diagram of health cloud service platform demand analysis for chronic diseases.

**Figure 2:** Basic framework of chronic disease health cloud service platform.

**Figure 3:** Data mining flow chart of chronic diseases in cloud service platform based on DT.

**Figure 4:** Flow chart of clustering analysis based on K-means algorithm.

**Figure 5:** Waveform diagram of pulse wave of original acquisition.

**Figure 6:** Pulse wave waveform processed by cloud platform DT.

**Figure 7:** EEG signal map of epileptic patients with original acquisition.

**Figure 8:** EEG signal map of epileptic patients processed by DT of cloud platform.

**Figure 9:** Statistics of age distribution of patients with epilepsy.

RETRACTED

**Figure 10:** Comparison of HAMA and HAMD scores in different groups. (a) HAMA comparison; (b) HAMD comparison) (^∗∗∗^indicates very significant difference compared with control group, *P* < 0.001).

**Figure 11:** Comparison of SCL-90 scores between two groups. (^∗∗^means clear distinction versus controls, *P* < 0.01).

**Figure 12:** Comparison of scores of different EPQ-RSC scales. (^∗^means obvious difference from controls, *P* < 0.05; ^∗∗^indicates clear distinction from controls, *P* < 0.01).

**Table 1:** Basic information table of patients.

Field name	Data type	Whether to type	Note
ID-code	int	Yes	Not null
Name	tinyint	No	Not null
Gender	varchar	No	Not null
Age	datetime	No	Not null
Occupation	varchar	No	Not null
Educational level	varchar	No	Not null
Contact way	varchar	Yes	Not null

**Table 2:** Medical history of patients.

Field name	Data type	Whether to type	Note
Medical history ID-code	int	Yes	Not null
Personal disease	varchar	No	Not null
Disease	varchar	Yes	Not null
Family member	varchar	No	Not null
Sign	varchar	Yes	Not null

**Table 3:** Patient disease diagnosis and treatment table.

Field name	Data type	Whether to type	Note
ID-code	int	No	Not null
Doctor ID	int	No	Not null
Date	Datetime	Yes	Not null
Inspection item	varchar	Yes	Not null
Diagnosis result	varchar	No	Not null
Treatment plan	varchar	Yes	Not null

**Table 4:** Patient assessment index.

Field name	Data type	Whether to type	Note
ID-code	int	Yes	Not null
Introduction of total evaluation index	varchar	No	Not null
Introduction of no obvious symptoms	varchar	No	Not null
Score range of no obvious symptoms	Numeric	Yes	Not null
Introduction of mild symptoms	varchar	No	Not null
Score range of mild symptoms	Numeric	Yes	Not null
Introduction of moderate symptoms	varchar	No	Not null
Score range of moderate symptoms	Numeric	Yes	Not null
Introduction of heavy symptoms	varchar	No	Not null
Score range of heavy symptoms	Numeric	Yes	Not null
Introduction of severe symptoms	varchar	No	Not null
Score range of severe symptoms	Numeric	Yes	Not null
Score	int	No	Not null

**Table 5:** Comparison of basic information between epilepsy group patients and control group.

Item	Epilepsy group	Control group	*P*
Age	50.35 ± 4.85	49.88 ± 5.67	0.258
Gender			0.219
Male	26 (61.90)	24 (60.00)	
** **Female	16 (38.10)	16 (40.00)	
Nationality [case (%)]			0.327
** **Han nationality	34 (80.95)	32 (80.00)	
** **Ethnic minorities	8 (19.05)	8 (20.00)	
Region (case (%))			0.256
** **Urban areas	25 (59.52)	24 (60.00)	
** **Rural areas	17 (40.48)	16 (40.00)	
Educational level			0.315
** **Primary school	8 (19.05)	8 (20.00)	
** **Junior high school	16 (38.10)	15 (37.50)	
** **University	11 (26.19)	10 (25.00)	
** **Graduate students and above	7 (16.67)	7 (17.50)	
Occupation			0.284
** **Cadres	8 (19.05)	9 (22.50)	
** **Teachers	5 (11.90)	6 (15.00)	
** **Workers	20 (47.62)	19 (47.50)	
** **Farmers	3 (7.14)	2 (5.00)	
** **Others	6 (14.29)	4 (10.00)	
Marital status			0.199
** **Married	33 (78.57)	32 (80.00)	
** **Unmarried	2 (4.76)	1 (2.50)	
** **Divorced or widowed	7 (16.67)	7 (17.50)	

RETRACTED

## Data Availability

The simulation experiment data used to support the findings of this study are available from the corresponding author upon request.
